RETRACTED

# A Machine-Learning-Based System for Prediction of Cardiovascular and Chronic Respiratory Diseases

**DOI:** 10.1155/2021/2621655

**Published:** 2021-11-01

**Authors:** Wajid Shah, Muhammad Aleem, Muhammad Azhar Iqbal, Muhammad Arshad Islam, Usman Ahmed, Gautam Srivastava, Jerry Chun-Wei Lin

**Affiliations:** ^1^Capital University of Science and Technology, Islamabad 44000, Pakistan; ^2^National University of Computer and Emerging Sciences (NUCES), Islamabad 44000, Pakistan; ^3^School of Computing and Artificial Intelligence, Southwest Jiaotong University, Chengdu 611756, China; ^4^Department of Computer Science,Electrical Engineering and Mathematical Sciences, Western Norway University of Applied Sciences, Bergen 5063, Norway; ^5^Department of Mathematics and Computer Science, Brandon University, Brandon, Canada; ^6^Research Centre for Interneural Computing, China Medical University, Taichung 40402, Taiwan

## Abstract

Cardiovascular and chronic respiratory diseases are global threats to public health and cause approximately 19 million deaths worldwide annually. This high mortality rate can be reduced with the use of technological advancements in medical science that can facilitate continuous monitoring of physiological parameters—blood pressure, cholesterol levels, blood glucose, etc. The futuristic values of these critical physiological or vital sign parameters not only enable in-time assistance from medical experts and caregivers but also help patients manage their health status by receiving relevant regular alerts/advice from healthcare practitioners. In this study, we propose a machine-learning-based prediction and classification system to determine futuristic values of related vital signs for both cardiovascular and chronic respiratory diseases. Based on the prediction of futuristic values, the proposed system can classify patients' health status to alarm the caregivers and medical experts. In this machine-learning-based prediction and classification model, we have used a real vital sign dataset. To predict the next 1–3 minutes of vital sign values, several regression techniques (i.e., linear regression and polynomial regression of degrees 2, 3, and 4) have been tested. For caregivers, a 60-second prediction and to facilitate emergency medical assistance, a 3-minute prediction of vital signs is used. Based on the predicted vital signs values, the patient's overall health is assessed using three machine learning classifiers, i.e., Support Vector Machine (SVM), Naive Bayes, and Decision Tree. Our results show that the Decision Tree can correctly classify a patient's health status based on abnormal vital sign values and is helpful in timely medical care to the patients.

RETRACTED

## 1. Introduction

The reliance on medical healthcare systems over technology can never be denied. Since the past several decades, innovations in technology have greatly benefited multifarious medical applications, especially in the fields of *diagnosis*, *risk assessment*, and *prognostication* [1]. Among different mechanisms in Computer-aided Medical Applications, Machine Learning (ML) plays a vital role in predicting certain conditions of patients, providing feasibility to doctors and caregivers to render treatment strategies accordingly [1, 2]. The prime purpose of initiating ML into medicines is to have reliable medical procedures for patients suffering from different chronic diseases [3]. Therefore, in the modern era, data- and model-driven intelligent and smart healthcare systems are required to be implemented to not only assist chronic disease patients but also concerned healthcare practitioners and caregivers.

According to the World Health Organization (WHO), cardiovascular and chronic respiratory diseases are the major causes of death globally [4, 5]. Every year, approximately 17.5 million people die due to cardiovascular diseases (CVDs) [1]; around 1.59 million people die because of chronic respiratory diseases [2]. The CVDs include heart attack, stroke, heart failure, arrhythmia, and heart valve problems [1], whereas asthma, occupational lung diseases, hypoxemia, and hypercapnic are chronic respiratory diseases [2]. Lack of sufficient capabilities of various healthcare systems hinders the process of disease curing. Thereby, the reliability of patients on the medical systems gets compromised [5]. An instant response to the critical condition of a patient is the consequential aspect that can benefit the doctors as well as the patients. In this regard, researchers across the globe are contributing their efforts to introduce intelligent and efficient mechanisms for medical healthcare systems to reduce the death risks caused by deadly diseases [6–9].

The contemporary state-of-the-art techniques assist the medical healthcare systems by predicting the contemporaneous state of a patient using several ML techniques like Naive Bayes, random forest, and neural networks [6, 7, 10]. These techniques employ the historical features of a patient to generate the corresponding health alerts. However, to the best of our knowledge, these techniques solely predict the real-time condition of a patient. None of them focuses on predicting the forthcoming situation of a patient. In intense medical situations, the condition of a patient could get worse within a fraction of a second [11, 12]. The average response times in critical situations are between 1 and 3 minutes [11, 13]. During this span, lack of adequate information regarding patients' conditions could present medical experts with a critical situation. We believe that predicting the forthcoming situation of a patient can play a pivotal role in rendering efficacious treatment. Also, predicting the patient's futuristic condition could help save lives and provide caregivers potential information to be contemplated. This study overcomes this issue by developing the cardiovascular and chronic respiratory diseases prediction system that predicts the forthcoming condition of a patient for the next 60 seconds and 3 minutes. The system forecasts the vital signs of chronic respiratory and cardiovascular diseases (i.e., heart failure, hypoxemic, and hypercapnic) and generates the corresponding health alerts (low heart rate or high heart rate, etc.). Thereafter, the condition of a patient is predicted by classifying these health alerts into 38 classes. The employed dataset contains a wide variety of patients' vital signs recorded under 32 surgical situations [12]. We have taken the assistance of medical experts to mark the most relevant vital signs against respective diseases (i.e., hypoxemic and hypercapnic, and heart failure), which ensued in 10 vital signs against each disease. Afterwards, the linear regression and polynomial regression with degrees 2, 3, and 4 are applied to these vital signs to forecast the vital signs for the next 60 seconds and 3 minutes. These regression models are trained using 50,000 to 100,000 samples of vital signs recorded within an interval of 10 milliseconds. These forecasted values are then assigned to SVM [14], Decision Tree [15], and Naive Bayes [16] classifiers to predict the upcoming condition of a patient. The results revealed that the decision tree had obtained commendable prediction results. These findings suggest that the proposed system has significant capability to predict the forthcoming situation of patients suffering from cardiovascular and chronic respiratory diseases. The specific contributions of this work are as follows:

- In-depth analysis of state-of-the-art techniques to identify the merits and demerits of several existing techniques related to vital signs and disease prediction
- A novel machine-learning-based prediction and classification system to provide futuristic values of the important vital signs for the two diseases and classify the patients' health situations
- In-depth experimental analysis to gauge the performance of several machine learning models for vital signs prediction and disease classification

The rest of the paper is organized as follows.  Section 2 presents an overview of contemporary state-of-the-art techniques.  Section 3 delineates the proposed methodology. The obtained results and their discussions are presented in Sections 4 and 5, respectively.  Section 6 presents the conclusions along with the future dimensions of the proposed study.

RETRACTED

## 2. Related Work

We have performed a comprehensive analysis of the literature that has led us to identify the existing gaps and to propose the appropriate solutions accordingly. A plethora of studies has employed different ML classification techniques to diagnose or predict different diseases and their symptoms. Let us scrutinize a few of them.

In Ref. [17], authors have presented a study to diagnose heart diseases, AIDS, brain cancer, diabetes, dengue, and hepatitis C. The machine-learning algorithms, Naive Bayes, J48, K-Nearest Neighbors, and C4.5 algorithms, have been employed to map the patients onto different classes of the above-stated diseases. The comparisons of the results among harnessed classifiers have revealed that C4.5 outperformed with 83.6% prediction accuracy, followed by J48 and Naive Bayes classifiers achieving 81.1% and 75.97% prediction accuracies, respectively. Similarly, in Ref. [18], coronary heart diseases have been diagnosed using Dichotomiser3 (ID3), Classification and Regression Tree (CART), and Decision Tree (DT) algorithms. The CART, DT, and ID3 have attained 83.49%, 82.50%, and 72.93% accurate prediction rates, respectively. The technique [10] predicts heart diseases, diabetes, and breast cancer using different machine-learning algorithms. The Naive Bayes algorithm has produced 74% accurate results in predicting heart diseases. For breast cancer prediction, the fuzzy decision tree algorithm has obtained high prediction accuracy as compared to C4.5 and ANN. The study [19] has classified healthy and Parkinson-infected people using SVM, Neural networks, Random Forest, Bagging and Boosting, ANN, KNN, and Naive Bayes models. The SVM has predicted Parkinson's disease with 99.49% accuracy. The ANN, KNN, and Naïve Bayes have produced 96.77%, 96.07%, and 74.31% prediction accuracies, respectively.

In another similar study [6], the potential of Naive Bayes and decision tree (J48) algorithms have been analyzed for predicting the survivability of patients diagnosed with lung cancer. Survivability is defined as someone who lives beyond five years post-disease period. The Naive Bayes and J48 have produced 92.37% and 94.43% accuracies, respectively. In Ref. [8], the dengue disease prediction model has been presented. The model has utilized Naive Bayes, Decision Tree (J48), Sequential Minimal Optimization (SMO), RANDOM Tree, and REP tree classifiers and produced 100%, 99.70%, 91.03%, and 75.60% accuracies, respectively.

RETRACTED

In Ref. [7], Intelligent Heart Disease Prediction Systems (IHDPS) have been designed using Decision Tree, Naïve Bayes, and Neural Network (NN) to predict different heart diseases. The system has extracted the hidden knowledge (patterns and relationships) associated with heart diseases by employing 15 different medical vital signs, such as age, sex, chest pain. The Naive Bayes, decision tree, and neural network algorithms have obtained 95%, 94.93%, and 93.54% prediction accuracies, respectively. In Ref. [9], authors have implemented the same model as of [10] to predict heart diseases using Decision Tree, J48, Logistic Model Tree (LMT), and Random Forest (RF) classifiers. In Ref. [20], Parkinson's disease has been predicted using symptoms-based features like olfactory loss and sleep disorder, etc. The study has employed Support Vector Machine (SVM) and Classification Tree (CT) classifiers. The SVM has outperformed with 85.48% prediction accuracy. In Ref. [21], the heart disease prediction model has been implemented using Naive Bayes, Decision Tree (DT), and KNN classifiers. The decision tree has attained 52% prediction accuracy, followed by KNN with 45.67% prediction accuracy. In a similar study [22], the predictive accuracies of Naive Bayes and decision tree classifiers have been compared on different medical datasets. For the lung cancer dataset, the decision tree and Naive Bayes classifiers have obtained 90.59% and 82.31% accuracies, respectively.

Similarly, various studies adopt different approaches based on machine learning or data mining to perform certain predictions about medical science [23–29]. However, to the best of our knowledge, none of the existing studies has focused on forecasting vital signs using regression models to predict the imminent condition of a patient. We believe that the prediction of forthcoming situations could substantially assist the medical experts in terms of taking immediate precautions and formulating an on-time treatment strategy. Moreover, the contemporary state-of-the-art technique lacks the prediction of vital signs for severe chronic diseases like hypoxemic and hypercapnic. Our study overcomes these issues by forecasting the vital signs for chronic respiratory diseases (i.e., hypoxemic and hypercapnic) using different regression models to predict the condition of patients for the next 60 seconds and 3 minutes using the dataset comprising 50,000 to 100,000 million samples of vital signs. From this extensive list of samples, we have exhaustively picked the relevant vital signs of chronic and cardiovascular diseases by taking the assistance of medical experts. The recapitulation illustrated in Table 1 coherently presents the main aspects of the contemporary state-of-the-art studies.

RETRACTED

Cardiovascular diseases can also result from hypertension, with 17 out of 67 causes of death caused by circulatory diseases [30]. The other 50 deaths are unlikely to be causal [30]. Biomarkers are also crucial for designing, developing, and better understanding cardiovascular disease [31]. The prognostic biomarker can help treat cardiovascular disease vital signs that include heart failure and coronary heart disease [31]. Different diseases are also treated as related to heart issues [32]. Rosacea was found to have risk factors associated with the heart. It is found that the cardiovascular disease patient should pay attention to inflammatory and metabolic disorders [32].

## 3. Methodology

Identifying the risk related to heart disease can help health facilities to decide which type of procedures or equipment is appropriate. This can help increase the mortality rate of humans. This research uses the forecasting and classification model to assess the patient's conditions suffering from cardiovascular (heart failure) and chronic respiratory (hypoxemia and hypercapnia) diseases. We used the real dataset for the patients and evaluated the vital signs for each distinct disease. Linear and polynomial regression models first use the vital signs to forecast the next one and three minutes' vital signs as mentioned in Figure 1. Then, by using the forecasted results, the classification models have been used according to low, normal, and high ranges of each distinct vital sign. The study has identified the hybrid model that uses the previous minute's data to forecast the vital signs and classify into the distinct label that helps the health worker make quick decisions. The research demonstrates that using the forecasting model with a combination of the time series data can help to produce high accuracy and substantially higher performance to related work. The model can detect potential hybrid regression models in predicting the imminent condition of the patient.

### 3.1. PMC TeleHealth System

The proposed system is a part of the *Patient Medical Condition TeleHealth* (PMC TeleHealth) system (Figure 2). The main purpose of the PMC TeleHealth system is to present the real-time medical condition of a patient in the form of *vital signs, visual charts*, *health alerts, etc.* The doctors or caregivers can then analyze this information to treat the patients accordingly. One of the critical components of the PMC TeleHealth system is the *Critical Condition Vital Signs (CCVS*) prediction system. The *CCVS* holds the responsibility for disease prediction. This study focuses on optimizing the CCVS in forecasting the future vital signs of severe diseases like hypoxemia, hypercapnic, and heart failure to meet the emerging demands of healthcare systems.

RETRACTED

### 3.2. Dataset

We have employed the dataset formulated by the *University of Queensland* [12]. It contains many vital signs for cardiovascular disease (i.e., heart failure) and cardiovascular diseases (i.e., hypoxemic and hypercapnic). These vital signs were captured via real-time monitoring of 32 different patients at the Royal Adelaide Hospital. The duration of data acquisition was 13 minutes to 5 hours. The pattern of vital signs recording followed the interval of 10 milliseconds, which produced 10 million vital signs samples in biomedical readings. The raw form of the acquired data file contained a total of 65 vital signs. We have taken the assistance of medical experts to mark the most relevant vital signs against the respective diseases. The chosen vital signs are shown in Table 2.

### 3.3. Preprocessing and Normalization

Since the raw file of the UQ dataset contains different surgical situations for a single patient in multiple files, we have converted them into a single file by omitting all the redundancies, such as null values or missing values. The raw dataset contains different files for a single patient, in which time continuation is a complex problem. Therefore, managing these files and their time continuation issues in a single file is a time-consuming effort. The dataset also contains null or missing values for different vital signs. These null values or missing values affect the experimental results. Therefore, we identified and removed the null values from the dataset and replaced the missing instances with an average of previous and next readings of the same vital sign value. Afterwards, the dataset was divided into two files. One file contains the readings for cardiovascular disease, and another contains the readings for chronic repository diseases. As the vital signs' readings were in the form of varying numeric ranges, these have been scaled down on the same range through normalization. Figures 3 and 4 present the data characteristics for the employed vital signs related to chronic respiratory and cardiovascular diseases. The data characteristics are presented in terms of *minimum value*, *maximum value*, *mean*, and *standard deviation*.

### 3.4. Vital Signs and Classes

The vital signs of both diseases have been associated with each output class based on the global ranges of vital signs [28]. These global ranges direct to three conditions of a patient, namely, *low*, *medium*, and *high.* The ranges of these conditions against the vital signs of both diseases are shown in Table 3. The output classes have been defined by combining each vital sign with the mentioned three conditions (as shown in Tables 4, and 5). If all the vital signs are in the low range, the corresponding output class will be *Low*. The *Low* label indicates the critical condition of a patient requiring immediate medical attention. The normal ranges specify that the condition of a patient is entirely normal. If more than one vital sign lies in the low range and all other vital signs lie in the normal range, the output class will be *Low* (i.e., Low HR). Similarly, the vital signs lying in the high ranges stipulate the critical situation adhering to urgent attention.

RETRACTED

### 3.5. Regression Models

Regression analysis explores the relationship between dependent and independent variables. The dependent variable is one whose value must be forecasted (i.e., the value of a vital sign in our case). In contrast, the independent variable is used to explain the dependent variable as an input. We have employed two regression models to forecast patients' vital signs for the next 60 seconds and 3 minutes. These time frames have been chosen because average response times in critical situations of a patient are 60 seconds and 3 minutes [11, 12]. The harnessed regression models include the following:

(a) Linear regression: it fits a line to a dataset of observations and then analyzes it to predict the unobserved values [33]. The formal description of linear regression is presented in
  (1) $$\begin{array}{c} y=\beta_{0}+\beta_{1}\times x, \end{array}$$
where *y* (dependent variable) is a function of *x, β*_*0*_ is the intercept, and *β*_*1i*_ is the slope or coefficient.
(b) Polynomial regression: in polynomial regression, the relationship between independent variable *x* and dependent variable *y* is modelled as an *n*^*th*^ degree polynomial in *x* [34]. To forecast the vital signs, we have applied polynomial regression with degrees 2, 3, and 4 on the vital signs' readings. The polynomial regression equations with degrees 2, 3, and 4 are shown in equations (2), (3), and (4), respectively.

For degree 2:

(2) $$\begin{array}{c} y=\beta_{0}\times x^{2}+\beta_{1}\times x+\beta_{2}. \end{array}$$

For degree 3:

(3) $$\begin{array}{c} y=\beta_{0}\times x^{3}+\beta_{1}\times x^{2}+\beta_{2}\times x+\beta_{3}. \end{array}$$

For degree 4:

(4) $$\begin{array}{c} y=\beta_{0}\times x^{4}+\beta_{1}\times x^{3}+\beta_{2}\times x^{2}+\beta_{3}\times x+\beta_{4}. \end{array}$$

### 3.6. Classification

Once all the vital signs have been forecasted, apply the earlier mentioned regression models. The next step involves their classification into 38 classes (i.e., 38 classes for cardiovascular disease and 38 classes for chronic respiratory diseases). As explained earlier, the contemporary state-of-the-art studies reveal that Support Vector Machine, Decision Tree, and Naive Bayes classifiers have produced promising results. Therefore, this study has also applied the same classifiers on the forecasted values of vital signs [8, 9, 19]. For vital medical signs, traditional classification models that achieved high performance are selected [19]. In addition, the data size is small. Then, traditional algorithms can perform better. The deep learning architectures required high-end infrastructure to train and predict in a reasonable time. Also, when there is a lack of data understanding or lack of domain knowledge, then deep learning models outshine as learning methods can develop their features. In our case, the vital signs' data with distinct characteristics can help to forecast and classify results. That is why we did not opt for the deep learning models.

RETRACTED

### 3.7. Evaluation

The standard evaluation measures, *precision*^33^, *recall*^33^, *f-measure*^33^, *mean square error*^34^, and *mean absolute percentage error*^35^, have been calculated to evaluate the performance of the proposed system. The evaluation results are explained in Section 4.

## 4. Experiments and Results

This section encompasses the results obtained by applying the methodology explained in Section 3. As explained earlier, we have split the vital signs' data for both the diseases and performed individual predictions for each category (i.e., cardiovascular and chronic respiratory) of disease.

### 4.1. Cardiovascular Disease Experimentation

#### 4.1.1. 60-Second Forecasted Vital Signs

To predict the future vital signs of cardiovascular disease (i.e., heart failure), the linear regression model and polynomial regression model with degrees 2, 3, and 4 have been trained on the samples of 50,000 vital signs having an interval of 10 milliseconds. After that, these trained models have been utilized to forecast future readings against each vital sign for the next 60 seconds.

- Classification using linear regression*:* the linear regression model has produced the best forecasted values for the Spo2 vital sign for the period of the next 60 seconds. The most negligible value of MAPE has been obtained against spo2 (i.e., the value of 3.29). Among all the classifiers, the Naïve Bayes has outperformed by predicting heart failure with an F-measure of 0.55. The obtained results against each classifier are illustrated in Table 6.
- Classification using polynomial regression (degree 2, 3, and 4): among all the polynomial regression models, the model built using degree 2 has outperformed others. The model has forecasted the vital signs for cardiovascular disease by producing a minimum value of MAPE up to 2.75 and a maximum value of MAPE up to 13.15. The Naive Bayes and decision tree classifiers have predicted heart failure with significant values of F-measure (i.e., 0.75 and 0.73). The polynomial regression with degree 3 has behaved almost identical to the polynomial regression model with degree 2 by achieving an F-measure of 0.72 for the Naïve Bayes classifier, whereas the polynomial regression model with degree 4 has predicted heart failure with the lowest value of *F*-measure (i.e., up to 0.51). The detailed results for an outperformed regression model are reported in Table 7.
- Classification using hybrid regression model:in the hybrid model, we have combined those regression models that have produced the least value for MAPE for a certain vital sign of heart failure disease. The best models and the corresponding vital sign and MSPE scores are shown in Table 8.
- Afterwards, these models have been combined to scrutinize the potential of their collective (i.e., hybrid) performance. Surprisingly, the hybrid model has not produced as promising results as the individual models. In the hybrid model, the highest obtained value of F-measure is 0.66, attained using the Naïve Bayes classifier. These outcomes yield that the hybrid approach cannot be deemed a quintessential approach in predicting heart failure for the next 60 seconds. The detailed results obtained using the hybrid model are shown in Table 9.

RETRACTED

#### 4.1.2. 3-Minute Forecasted Vital Signs

In Section 4.1.1, we have already explained the process related to forecasting vital signs for the 1-minute bracket. A similar process is employed to forecast vital signs for 3 minutes time unit and further explained below. The details regarding the selection of these time frames have already been explained in Section 3.

- Classification using linear regression: when the linear regression model has been applied to forecast the vital signs for the next 3 minutes, all the classifiers (i.e., SVM, Naïve Bayes, and decision tree) have predicted the heart failure with moderate values of F-measure. The Naïve Bayes classifier has achieved an F-measure of 0.39 followed by SVM and decision tree with F-measures of 0.35 and 0.19, respectively. However, the model has not performed well in terms of MAPE (i.e., it has produced a significant value of MAPE compared to the preceding models). The detailed results against each classifier are reported in Table 10.
- Classification using polynomial regression (degrees 2, 3, and 4): to predict heart failure disease for the next 3 minutes using polynomial regression models, similar behaviour has been observed as the next 1-minute prediction. The polynomial regression model with degree 2 has performed comparatively better than the polynomial regression models with degrees 3 and 4. The model has predicted heart failure with MAPE scores from 3.19 to 15.93. Among all the classifiers, the decision tree has obtained the highest value of F-measure (i.e., 0.75). Contrary to the best cardiovascular prediction model for the next 1 minute (i.e., linear regression), the best model is polynomial regression with degree 2. As the degrees of the polynomial regression model have become higher (i.e., 3 and 4), the performance of prediction models started to decline. The polynomial regression model with degree 3 has obtained the MAPE scores from 32.99 to 952.04. The best value of F-measure is 0.55, which has been obtained using the Naïve Bayes classifier. For polynomial regression with degree 4, all the classifiers have obtained the values of F-measure around 0.37. The detailed results for the best prediction model are presented in Table 11.
- Hybrid regression model: to find the best combination of regression techniques, we have picked the regression models with the least MAPE value. The best regression models, along with the corresponding vital signs, are shown in Table 12.

RETRACTED

The hybrid model for predicting heart failure for the next 3 minutes has performed better than the hybrid model for 60-second prediction. It has obtained the least error values than the linear regression model and polynomial regression models. In the hybrid model, the best score of F-measure is 0.60, which has been obtained through the Naïve Bayes classifier. The detailed results for 3-minutes predictions using the hybrid model are shown in Table 13.

### 4.2. Chronic Respiratory Disease Experimentation

In this section, we discuss the forecasting and classification of chronic respiratory disease. For each vital sign, a separate model is developed, evaluated, and compared. The high accurate results are then selected to classify the vital sign based on its time series forecasted values. The following section presents the forecasted 60 and 180 seconds. Then, we explained the classification results.

#### 4.2.1. 60-Second Forecasted Vital Signs

Similar to 60-second forecasted vital signs for cardiovascular disease, to forecast the future vital signs for chronic respiratory diseases (i.e., hypoxemic and hypercapnic), all the regression models (i.e., linear regression, polynomial regression (degree 2, 3, and 4) have been trained on 50,000 samples of vital signs having ten millisecond intervals among them. These trained models have been then employed to forecast the vital signs for the next 60 seconds. After that, the classification has been performed on these forecasted values.

- Classification using linear regression: the classification results against a linear regression model to predict a patient's condition for the next 60 seconds are unsatisfactory. All the classifiers have obtained very low *F*-measure scores. The obtained values for all classifiers, MSE, and MAPE scores of the linear regression model are shown in Table 14.
- Classification using polynomial regression (degree 2, 3, and 4): in the polynomial regression model with degree 2, the Naive Bayes classifier has obtained an F-measure of 0.23, and the vital sign SPO2 has obtained the mean square error of 1.09. Compared to the linear regression, the value of the F-measure has slightly improved (i.e., from 0.13 to 0.23). The results are shown in Table 15.
- The polynomial regression model with degree 3 has attained the F-measure of 0.30, an improved score than the F-measure of degree 2 models. In the case of a polynomial regression model with degree 4, the F-measure scores of all the classifiers have receded. These outcomes demonstrate that the polynomial regression model with degree 3 could be employed to predict the next 60-second condition of a patient suffering from hypoxemic and hypercapnic diseases with adequate accuracy.
- Classification using the hybrid regression model: to find the best combination of regression models, we have picked the regression models with the least values of MAPE. The best models are shown in Figure 5.

RETRACTED

All of these models have been combined to analyze their performance in a hybrid manner. To predict the condition of a chronic respiratory patient for the next 60 seconds, all the classifiers in the hybrid model have achieved the values of *F*-measures around 0.20, which are quite lower than the F-measure scores of the previous models. The detailed results of the hybrid model are shown in Table 16.

#### 4.2.2. 3-Minute Forecasted Vital Signs

The exact process of forecasting the vital signs of chronic respiratory diseases for the next 60 second (see Section 4.2.1) has been repeated to forecast the vital signs of chronic respiratory diseases for the next 3 minutes.

- Classification using linear regression:when the linear regression model has been employed on 3-minute forecasted vital signs, the Naive Bayes classifier has achieved the high value of *F*-measure (up to 0.24). The results are shown in Table 17.
- Classification using polynomial regression (degree 2, 3, and 4):the polynomial regression model with degree 2 has obtained very low values of *F*-measures against all the classifiers (i.e., values around 0.04). For polynomial regression with degree 3, the attained value of the *F*-measure is much better than the *F*-measure of the degree 2 models (i.e., 0.20 vs. 0.04). The polynomial regression model with degree 3 has attained identical poor performance as of degree 2 models. The obtained values against each classifier for the best-performing model are shown in Table 18.
- Classification using the hybrid regression model: to find the best combination of regression models, the models with the lowest MAPE values have been chosen. The employed models and corresponding vital signs are shown in Figure 6.

RETRACTED

When these top regression models have been combined, the decision tree classifiers have obtained the result by scoring an F-measure of 0.11. So far, this hybrid model has achieved the worst values of F-measure. The detailed results are reported in Table 19.

## 5. Results and Discussion

- Regression techniques: let us recapitulate and analyze the obtained results against each proposed prediction model. The potential of the regression technique could be better described by contemplating the corresponding value of mean absolute percentage error. The mean absolute percentage error (MAPE) determines the prediction accuracy of a forecasting model.  Table 20 presents MAPE scores for each regression model along with the respective vital signs. Overall, the linear regression model has performed well in forecasting the vital signs of cardiovascular disease in the next 60 seconds, and the polynomial regression models have performed well in forecasting the vital signs for the next 3 minutes.
- Classification techniques: to classify a patient's condition into 38 classes, we have opted for Naive Bayes, support vector machine, and decision tree classifiers. All the classification techniques have been evaluated using standard evaluation measures (i.e., precision, recall, and F-measure). Since the F-measure is the harmonic mean of precision and recall, overall classification results have been assessed based on F-measure.  Table 21 illustrates the obtained values of evaluation measures. In Table 21, the yellow boxes indicate the best scores of evaluation measures, whereas the boxes with pink shade determine the poor values of evaluation measures.

Table 21 shows the performance of each harnessed classifier. The prediction score of precision, recall, and F-measures obtained from the Naïve Bayes, SVM, and Decision Tree for a heart failure patient for the next 60 seconds are {0.72, 0.82, 0.75}, {0.67, 0.60, 0.61}, and {0.80, 0.76, 0.73}, respectively. This means we can use either Naïve Bayes or a decision tree to predict the heart failure patient for the next 60 seconds. Similarly, for Chronic Respiratory patients, the precision, recall, and F-measure for the next 60 seconds are {0.30, 0.29, 0.28}, {0.30, 0.27, 0.28}, and {0.31, 0.31, 0.30}, respectively. These results show that the Decision Tree is highly recommended for chronic respiratory disease prediction. The prediction score of precision, recall, and F-measures obtained from the Naïve Bayes, SVM, and Decision Tree for heart failure patients for next 3 minutes are {0.59, 0.67, 0.60}, {0.73, 0.51, 0.53}, and {0.78, 0.76, 0.75}, respectively. This means that we can use a decision tree for predicting the plight of the heart failure patient for the next 3 minutes. Similarly, for the Chronic Respiratory patients, the precision, recall, and F-measure for the next 3 minutes are {0.25, 0.26, 0.24}, {0.23, 0.17, 0.18}, and {0.21, 0.20, 0.20}. These results show that either Naïve Bayes or Decision Tree is recommended for the prediction of chronic respiratory diseases (for the next 3 minutes values of vital signs).

RETRACTED

Overall, the performance of the decision tree has remained consistent in all the scenarios. The best classification results have been attained in predicting the condition of a cardiovascular patient for the next 60 seconds. The Naïve Bayes and Decision Tree have produced the highest values of precision, recall, and *F*-measure for predicting cardiovascular disease (i.e., heart failure) for the periods of the upcoming 60 seconds and 3 minutes. However, the classification of chronic respiratory diseases has not yielded many promising results. Based on this analysis, we claim that the proposed system holds sufficient potential in predicting the condition of cardiovascular patients in foreseeing critical periods (i.e., 60 seconds and 3 minutes).

Figures 3 and4 show the statistical insight (*Min*, *Mean*, *Max*, and *Standard Deviation*) of the vital signs available in the dataset. All measures except standard deviation are presented in terms of a binary logarithm. In CVD Figure 4, all vital signs have a relatively high standard deviation except SpO2. It is noteworthy that a standard deviation of NBP (Sys) is exceptionally high. In CRD Figure 3, imCO2 among the four additional vital signs has the lowest standard deviation, and etO2 and inO2 show exceptionally high standard deviation.

## 6. Conclusions

Cardiovascular and chronic respiratory diseases are some of the issues faced by health care. Due to the time-independent lifestyle, both diseases affect mortality across the globe. Heart attack occurs without any apparent symptoms. An intelligent method is utilized to forecast the vital signs that might help save the patient with cardiovascular and chronic respiratory disease. The computer-aided system may prevent or mitigate heart attacks and help in reducing the mortality rate. The effective identification of the machine-learning model concerning data is a challenging task. In this paper, we have discussed the details of predicted models for the forecasting of vital sign values that are ultimately helpful for the realization of a machine-learning-based system for the prediction of chronic diseases. This study also aims to facilitate caregivers and medical experts to provide in-time medical assistance to the patients to reduce the fatality rate due to cardiovascular and chronic respiratory complications in indoor patients, particularly after surgical procedures. It is necessary to assess the appropriateness of the prediction model according to the nature of the data.

RETRACTED

In summary, key findings from this work include evidence of the effectiveness of polynomial regression for the prediction of the vital signs that shows the curvilinear nature of the vital signs used in this study. We have fulfilled the requirement of employing a sizeable comprehensive dataset to build confidence in the polynomial regression prediction model. In addition, the prediction outcomes are used to train the classifiers to identify the state of the patient. Our results show that the Decision Tree can correctly classify the condition of the patient. Decision-Tree-based classifiers are generally considered intuitive. They do not require an accumulation of multiple variables; however, their use under the practical restraints of missing data must be critically analyzed.

## Figures and Tables

**Figure 1:** Schematic diagram of the proposed methodology for predicting CVD and CRDs.

**Figure 2:** Generic PMC TeleHealth system framework.

**Figure 3:** Data characteristics of vital signs related to chronic respiratory disease.

**Figure 4:** Data characteristics of vital signs related to cardiovascular disease.

**Figure 5:** Best regression models for 60-second forecasted vital signs.

**Figure 6:** Best regression models for 3-minute forecasted vital signs.

**Table 1:** Summarized results of contemporary state-of-the-art techniques.

Year	Data description	Approaches	Accuracy (%)
Reference [19], 2015	Parkinson's disease dataset	SVM	99.49
		ANN	96.77
		KNN	96.07
		Decision Tree	95
		Random Forest	90.26
		Naive Bayes	74.31
Reference [8], 2015	Dengue dataset	Naive Bayes	100
Reference [9], 2015	Cleveland database of UCI repository	Decision Tree (J48)	56.76
Reference [20], 2014	Parkinson's disease dataset	SVM	85.48
Reference [22], 2013	Lung cancer dataset	Decision Tree	90.59
	Heart dataset	Naive Bayes	80.75
	Dermatology	Naive Bayes	82.32
Reference [17], 2013	Cancer	Decision Tree	97.77
	Blood bank sector	J48	89.9
	Diabetes mellitus	C4.5	82.6
	HIV/AIDS	C4.5	81.8
	Tuberculosis	KNN	78
	Hepatitis C	Decision Rule	73.20
	Heart disease	Naive Bayes	60
Reference [10], 2013	Heart disease	Naive Bayes	74
Reference [18], 2013	Heart disease dataset (Cleveland Clinic Foundation)	CART	83.49
Reference [7], 2013	Cleveland Heart Disease database	Naive Bayes	95
Reference [6], 2012	Lung cancer (SEER dataset)	Decision Tree (C4.5)	94.43
Reference [21], 2010	Heart disease dataset	Naive Bayes	52.33

RETRACTED

**Table 2:** Vital signs for CVD and CRDs.

Index	Vital sign	Index	Vital sign
1	HR	6	SpO2
2	SpO2	7	imCO2
3	NBP (Sys)	8	etCO2
4	NBP (Dia)	9	etO2
5	NBP (mean)	10	inO2

**Table 3:** Range of vital sign values (low, normal, and high).

Vital sign	Low ranges	Normal ranges	High ranges
spo2	Less than 94	Between 94 and 100	Greater than 100
etCO2	Less than 30	Between 30 and 43	Greater than 43
imCO2	Less than 1	Between 1 and 20	Greater than 20
etO2	Less than 60	Between 60 and 90	Greater than 90
inO2	Less than 60	Between 60 and 90	Greater than 90
HR	Less than 60	Between 60 and 100	Greater than 100
NBP (Sys)	Less than 100	Between 100 and 130	Greater than 130
NBP (Dia)	Less than 60	Between 60 and 90	Greater than 90

**Table 4:** Thirty-eight output classes for cardiovascular disease.

Class ID	Class label
1	Low
2	Normal
3	High
4	Low HR
5	Low spO2
6	Low NBP (Sys)
7	Low NBP (Dia)
8	Low HR, spO2
9	Low HR, NBP (Sys)
10	Low HR, NBP (Dia)
11	Low spO2, NBP (Sys)
12	Low spO2, NBP (Dia)
13	Low NBP (Sys), NBP (Dia)
14	Low HR, spO2, NBP (Sys)
15	Low HR spO2, NBP (Dia)
16	Low HR NBP (Sys), NBP (Dia)
17	Low spO2 NBP (Sys), NBP (Dia)
18	Low HR spO2, NBP (Sys), NBP (Dia)
19	High HR
20	High spO2
21	High NBP (Sys)
22	High NBP (Dia)
23	High HR spO2
24	High HR, NBP (Sys)
25	High HR, NBP (Dia)
26	High spO2, NBP (Sys)
27	High spO2 NBP (Dia)
28	High NBP (Sys) NBP (Dia)
29	High HR spO2, NBP (Sys)
30	High HR spO2 NBP (Dia)
31	High HR, NBP (Sys), NBP (Dia)
32	High spO2 NBP (Sys),NBP (Dia)
33	High HR spO2, NBP (Sys), NBP (Dia)
34	High HR low NBP (Sys), NBP (Dia)
35	High HR low NBP (Dia)
36	Low HR high NBP (Sys), NBP (Dia)
37	Low HR high NBP (Sys)
38	Low SPO2 high NBP (Sys)

**Table 5:** Thirty-eight output classes for chronic respiratory diseases.

Class ID	Class label
1	Low
2	Normal
3	High
4	Low spO2
5	Low etCO2
6	Low imCO2
7	Low etO2
8	Low inO2
9	High etCO2
10	High spO2
11	High imCO2
12	High etO2
13	High inO2
14	Low etCO2, spO2
15	Low etCO2, imCO2
16	Low etCO2, etO2
17	Low spO2, imCO2
18	Low spO2, etO2
19	Low imCO2, etO2
20	Low etCO2, spO2,imCO2
21	Low etCO2, spO2,etO2
22	Low etCO2,imCO2,etO2
23	Low spO2, imCO2,etO2
24	Low etCO2, spO2,imCO2, etO2
25	High etCO2, spO2
26	High etCO2, imCO2
27	High etCO2, etO2
28	High spO2, imCO2
29	High spO2, etO2
30	High imCO2, etO2
31	High etCO2, spO2,imCO2
32	High etCO2, spO2,etO2
33	High etCO2, imCO2,etO2
34	High spO2, imCO2,etO2
35	High etCO2, spO2,imCO2, etO2
36	High etCO2 low imCO2,etO2
37	High etCO2, low etO2
38	Low etCO2 high imCO2, etO2

RETRACTED

**Table 6:** Classification of CVD on 60-second forecasted vital signs using linear regression.

Classifier		Linear regression		Performance metrics		
	Vital sign	MSE	MAPE	Precision	Recall	*F*-measure
Naïve Bayes	spo2	**3.42738**	**3.29088**	0.52	0.62	0.55
	HR	42.21474	6.15772			
	NBP (Sys)	514.2794	16.94344			
	NBP (Dia)	87.87894	9.8375			
	NBP (mean)	133.2341	11.76452			
Support Vector Machine	spo2	**3.42738**	**3.29088**	0.47	0.52	0.49
	HR	42.21474	6.15772			
	NBP (Sys)	514.2794	16.94344			
	NBP (Dia)	87.87894	9.8375			
	NBP (mean)	133.2341	11.76452			
Decision Tree (J48)	spo2	**3.42738**	**3.29088**	0.32	0.42	0.35
	HR	42.21474	6.15772			
	NBP (Sys)	514.2794	16.94344			
	NBP (Dia)	87.87894	9.8375			
	NBP (mean)	133.2341	11.76452			

**Table 7:** Classification of CVD on 60-second forecasted vital signs using polynomial regression degree 2.

Classifier		Polynomial degree 2		Performance metrics		
	Vital sign	MSE	MAPE	Precision	Recall	*F*-measure
Naïve Bayes	spo2	**7.26112**	3.85538	0.72	0.82	0.75
	HR	7.9457	**2.75838**			
	NBP (Sys)	288.3866	13.15938			
	NBP (Dia)	79.68692	6.6934			
	NBP (mean)	84.37498	8.22226			
Support Vector Machine	spo2	**7.26112**	3.85538	0.67	0.60	0.61
	HR	7.9457	**2.75838**			
	NBP (Sys)	288.3866	13.15938			
	NBP (Dia)	79.68692	6.6934			
	NBP (mean)	84.37498	8.22226			
Decision Tree (J48)	spo2	**7.26112**	3.85538	0.80	0.76	0.73
	HR	7.9457	**2.75838**			
	NBP (Sys)	288.3866	13.15938			
	NBP (Dia)	79.68692	6.6934			
	NBP (mean)	84.37498	8.22226			

**Table 8:** Best regression models for 60-second forecasted vital signs.

Best model	Vital sign	MAPE
Linear regression	spo2	3.29
Polynomial degree 2	HR	2.75
Polynomial degree 3	NBP (Sys)	7.71
Polynomial degree 3	NBP (Dia)	6.76
Polynomial degree 3	NBP (mean)	6.99

**Table 9:** Hybrid classification for CVD on 60-second forecasted vital signs.

Classifier		Best settings		Performance metrics		
	Vital sign	MSE	MAPE	Precision	Recall	*F*-measure
Naïve Bayes	spo2	**3.49538**	**1.49338**	0.77	0.64	0.66
	HR	7.9457	2.75838			
	NBP (Sys)	83.08452	7.7184			
	NBP (Dia)	35.41272	6.76452			
	NBP (mean)	36.2189	6.99832			
Support Vector Machine	spo2	**3.49538**	**1.49338**	0.69	0.56	0.60
	HR	7.9457	2.75838			
	NBP (Sys)	83.08452	7.7184			
	NBP (Dia)	35.41272	6.76452			
	NBP (mean)	36.2189	6.99832			
Decision Tree (J48)	spo2	**3.49538**	**1.49338**	0.58	0.36	0.37
	HR	7.9457	2.75838			
	NBP (Sys)	83.08452	7.7184			
	NBP (Dia)	35.41272	6.76452			
	NBP (mean)	36.2189	6.99832			

RETRACTED

**Table 10:** Classification of CVD on 3-minute forecasted vital signs using linear regression.

Classifier		Linear regression		Performance metrics		
	Vital sign	MSE	MAPE	Precision	Recall	*F*-measure
Naïve Bayes	spo2	**4.56966**	**3.46076**	0.40	0.43	0.39
	HR	66.19176	8.4793			
	NBP (Sys)	615.8491	19.53128			
	NBP (Dia)	158.5331	15.1971			
	NBP (mean)	205.1541	15.85418			
Support Vector Machine	spo2	**4.56966**	**3.46076**	0.37	0.39	0.35
	HR	66.19176	8.4793			
	NBP (Sys)	615.8491	19.53128			
	NBP (Dia)	158.5331	15.1971			
	NBP (mean)	205.1541	15.85418			
Decision Tree (J48)	spo2	**4.56966**	**3.46076**	0.21	0.24	0.19
	HR	66.19176	8.4793			
	NBP (Sys)	615.8491	19.53128			
	NBP (Dia)	158.5331	15.1971			
	NBP (mean)	205.1541	15.85418			

**Table 11:** Classification of CVD on 3-minute forecasted vital signs using polynomial degree 2.

Classifier		Polynomial degree 2		Performance metrics		
	Vital sign	MSE	MAPE	Precision	Recall	*F*-measure
Naïve Bayes	spo2	**19.6604**	**4.66122**	0.59	0.67	0.60
	HR	9.87616	3.19928			
	NBP (Sys)	342.3416	15.93054			
	NBP (Dia)	186.2163	14.37694			
	NBP (mean)	170.2237	13.48256			
Support Vector Machine	spo2	**19.6604**	**4.66122**	0.73	0.51	0.53
	HR	9.87616	3.19928			
	NBP (Sys)	342.3416	15.93054			
	NBP (Dia)	186.2163	14.37694			
	NBP (mean)	170.2237	13.48256			
Decision Tree (J48)	spo2	**19.6604**	**4.66122**	0.78	0.76	0.75
	HR	9.87616	3.19928			
	NBP (Sys)	342.3416	15.93054			
	NBP (Dia)	186.2163	14.37694			
	NBP (mean)	170.2237	13.48256			

**Table 12:** Best regression models for 3-minute forecasted vital signs.

Best model	Vital sign	MAPE
Linear regression	spo2	3.46
Polynomial degree 2	HR	3.19
Polynomial degree 2	NBP (Sys)	15.93
Polynomial degree 2	NBP (Dia)	14.37
Polynomial degree 2	NBP (mean)	13.48

**Table 13:** Hybrid classification for CVD on 3-minute forecasted vital signs.

Classifier		Best settings		Performance metrics		
	Vital sign	MSE	MAPE	Precision	Recall	*F*-measure
Naïve Bayes	spo2	**4.63774**	**1.6672**	0.59	0.65	0.60
	HR	9.87616	3.19928			
	NBP (Sys)	342.3416	15.93054			
	NBP (Dia)	186.2163	14.37694			
	NBP (mean)	170.2237	13.48256			
Support Vector Machine	spo2	**4.63774**	**1.6672**	0.73	0.51	0.52
	HR	9.87616	3.19928			
	NBP (Sys)	342.3416	15.93054			
	NBP (Dia)	186.2163	14.37694			
	NBP (mean)	170.2237	13.48256			
Decision Tree (J48)	spo2	**4.63774**	**1.6672**	0.58	0.56	0.55
	HR	9.87616	3.19928			
	NBP (Sys)	342.3416	15.93054			
	NBP (Dia)	186.2163	14.37694			
	NBP (mean)	170.2237	13.48256			

**Table 14:** Classification of CRDs on 60-second forecasted vital signs using linear regression.

Classifier		Linear regression		Performance metrics		
	Vital sign	MSE	MAPE	Precision	Recall	*F*-measure
Naïve Bayes	spo2	**13.36**	**2.28019**	0.20	0.11	0.13
	etCO2	103.73	33.36002			
	imCO2	157.6569	57.40156			
	etO2	139.6594	13.53372			
	inO2	268.6022	19.60382			
Support Vector Machine	spo2	**13.36**	**2.28019**	0.00	0.00	0.00
	etCO2	103.73	33.36002			
	imCO2	157.6569	57.40156			
	etO2	139.6594	13.53372			
	inO2	268.6022	19.60382			
Decision Tree	spo2	**13.36**	**2.28019**	0.00	0.00	0.00
	etCO2	103.73	33.36002			
	imCO2	157.6569	57.40156			
	etO2	139.6594	13.53372			
	inO2	268.6022	19.60382			

RETRACTED

**Table 15:** Classification of CRDs on 60-second forecasted vital signs using polynomial regression degree 2.

Classifier		Polynomial degree 2		Performance metrics		
	Vital sign	MSE	MAPE	Precision	Recall	*F*-measure
Naïve Bayes	spo2	**2.3466**	**1.09438**	0.22	0.25	0.23
	etCO2	42.46008	22.48736			
	imCO2	68.92556	46.9466			
	etO2	137.1689	10.14428			
	inO2	328.6665	21.34718			
Support Vector Machine	spo2	**2.3466**	**1.09438**	0.21	0.22	0.20
	etCO2	42.46008	22.48736			
	imCO2	68.92556	46.9466			
	etO2	137.1689	10.14428			
	inO2	328.6665	21.34718			
Decision Tree (J48)	spo2	**2.3466**	**1.09438**	0.21	0.24	0.22
	etCO2	42.46008	22.48736			
	imCO2	68.92556	46.9466			
	etO2	137.1689	10.14428			
	inO2	328.6665	21.34718			

**Table 16:** Hybrid classification for CRDs on 60-second forecasted vital signs.

Classifier		Best setting		Performance metrics		
	Vital sign	MSE	MAPE	Precision	Recall	*F*-measure
1. Naïve Bayes	spo2	**2.3466**	**1.09439**	0.20	0.20	0.20
	etCO2	85.3974	20.55036			
	imCO2	68.92556	46.9466			
	etO2	89.73446	7.99454			
	inO2	268.6022	19.60382			
2. Support Vector Machine	spo2	**2.3466**	**1.09439**	0.24	0.17	0.19
	etCO2	85.3974	20.55036			
	imCO2	68.92556	46.9466			
	etO2	89.73446	7.99454			
	inO2	268.6022	19.60382			
3. Decision Tree (J48)	spo2	**2.3466**	**1.09439**	0.29	0.17	0.21
	etCO2	85.3974	20.55036			
	imCO2	68.92556	46.9466			
	etO2	89.73446	7.99454			
	inO2	268.6022	19.60382			

**Table 17:** Classification of CRDs on 3-minute forecasted vital signs using linear regression.

Classifier		Linear regression		Performance metrics		
	Vital sign	MSE	MAPE	Precision	Recall	*F*-measure
Naïve Bayes	spo2	**2.8818**	**1.33644**	0.25	0.26	0.24
	etCO2	53.82438	19.25942			
	imCO2	241.6078	33.53168			
	etO2	314.453	33.5174			
	inO2	336.4857	27.62782			
Support Vector Machine	spo2	**2.8818**	**1.33644**	0.01	0.05	0.02
	etCO2	53.82438	19.25942			
	imCO2	241.6078	33.53168			
	etO2	314.453	33.5174			
	inO2	336.4857	27.62782			
Decision Tree (J48)	spo2	**2.8818**	**1.33644**	0.16	0.19	0.17
	etCO2	53.82438	19.25942			
	imCO2	241.6078	33.53168			
	etO2	314.453	33.5174			
	inO2	336.4857	27.62782			

RETRACTED

**Table 18:** Classification of CRDs on 3-minute forecasted vital signs using polynomial regression degree 2.

Classifier		Polynomial degree 2		Performance metrics		
	Vital sign	MSE	MSPE	Precision	Recall	*F*-measure
Naïve Bayes	spo2	**2.57998**	**1.26394**	0.02	0.07	0.03
	etCO2	104.7052	27.64572			
	imCO2	96.76128	39.98942			
	etO2	182.6932	16.6988			
	inO2	330.6127	14.02962			
Support Vector Machine	spo2	**2.57998**	**1.26394**	0.03	0.08	0.04
	etCO2	104.7052	27.64572			
	imCO2	96.76128	39.98942			
	etO2	182.6932	16.6988			
	inO2	330.6127	14.02962			
Decision Tree (J48)	spo2	**2.57998**	**1.26394**	0.04	0.05	0.04
	etCO2	104.7052	27.64572			
	imCO2	96.76128	39.98942			
	etO2	182.6932	16.6988			
	inO2	330.6127	14.02962			

**Table 19:** Hybrid classification for CRDs on 3-minute forecasted vital signs.

Classifier		Polynomial degree 2		Performance metrics		
	Vital sign	MSE	MAPE	Precision	Recall	*F*-measure
Naïve Bayes	spo2	**2.57998**	**1.26394**	0.11	0.05	0.04
	etCO2	700.1815	78.09214			
	imCO2	96.76126	39.98942			
	etO2	3158.258	98.19944			
	inO2	334.8831	27.5847			
Support Vector Machine	spo2	**2.57998**	**1.26394**	0.14	0.09	0.06
	etCO2	700.1815	78.09214			
	imCO2	96.76126	39.98942			
	etO2	3158.258	98.19944			
	inO2	334.8831	27.5847			
Decision Tree (J48)	spo2	**2.57998**	**1.26394**	0.09	0.16	0.11
	etCO2	700.1815	78.09214			
	imCO2	96.76126	39.98942			
	etO2	3158.258	98.19944			
	inO2	334.8831	27.5847			

**Table 20:** Combined results of 4 regression techniques with heart failure and CRD.

Vital sign	Cardiovascular time = 60 seconds		Cardiovascular time = 180 seconds		Vital sign	Chronic respiratory time = 60 seconds		Chronic respiratory time = 180 seconds	
	Model	MAPE	Model	MAPE		Model	MAPE	Model	MAPE
SpO2	Linear regression	3.29	Linear regression	**3.46**	SpO2	Polynomial degree 2	**1.09**	Polynomial degree 2	**1.26**
Heart rate	Polynomial degree 2	2.75	Polynomial degree 2	3.19	etCO2	Polynomial degree 4	20.55	Linear regression	19.25
NBP (sys)	Polynomial degree 3	7.71	Polynomial degree 2	15/.93	imCO2	Polynomial degree 2	46.94	Linear regression	33.53
NBP (dia)	Polynomial degree 3	6.76	Polynomial degree 2	14.37	etO2	Polynomial degree 4	7.99	Polynomial degree 2	16.69
NBP (mean)	Polynomial degree 3	6.99	Polynomial degree 2	13.48	inO2	Linear regression	19.60	Polynomial degree 2	14.02

**Table 21:** Combined results using three classification techniques for heart failure and CRD.

CT	RM	Performance metrics heart failure in 60 seconds			Performance metrics chronic respiratory in 60 seconds			Performance metrics heart failure in 3 minutes			Performance metrics chronic respiratory in 3 minutes		
		Pre	Rec	FM	Pre	Rec	FM	Pre	Rec	FM	Pre	Rec	FM
NB	LR	0.52	0.62	0.55	0.20	0.11	0.13	0.40	0.43	0.39	0.25	0.26	0.24
	PN2	0.72	0.82	0.75	0.22	0.25	0.23	0.59	0.67	0.60	0.02	0.07	0.03
	PN3	0.77	0.70	0.72	0.30	0.29	0.28	0.77	0.46	0.55	0.20	0.11	0.13
	PN4	0.82	0.45	0.51	0.21	0.18	0.19	0.65	0.27	0.31	0.11	0.05	0.04
	H.A	0.77	0.64	0.66	0.20	0.20	0.20	0.59	0.65	0.60	0.11	0.05	0.04
SVM	LR	0.47	0.52	0.49	0.00	0.00	0.00	0.37	0.39	0.35	0.01	0.05	0.02
	PN2	0.67	0.60	0.61	0.21	0.22	0.20	0.73	0.51	0.53	0.03	0.08	0.04
	PN3	0.72	0.51	0.58	0.30	0.27	0.28	0.52	0.35	0.37	0.23	0.17	0.18
	PN4	0.68	0.51	0.51	0.20	0.06	0.09	0.56	0.39	0.37	0.14	0.09	0.06
	H.A	0.69	0.56	0.60	0.24	0.17	0.19	0.73	0.51	0.52	0.14	0.09	0.06
DT	LR	0.32	0.42	0.35	0.00	0.00	0.00	0.21	0.24	0.19	0.16	0.19	0.17
	PN2	0.80	0.76	0.73	0.21	0.24	0.22	0.78	0.76	0.75	0.04	0.05	0.04
	PN3	0.78	0.53	0.55	0.31	0.31	0.30	0.79	0.25	0.32	0.21	0.20	0.20
	PN4	0.82	0.39	0.45	0.20	0.08	0.09	0.67	0.24	0.28	0.08	0.10	0.08
	H.A	0.58	0.36	0.37	0.29	0.17	0.21	0.58	0.56	0.55	0.09	0.16	0.11

^*∗*^CT = classification techniques, RM = Regression Model, NB=Naïve Bayes, SVM=Support Vector Machine, DT = Decision Tree, LR = linear regression, PN2 = polynomial degree 2, PN3 = polynomial degree 3, PN4=polynomial degree 4, HA=hybrid approach, Pre = precision, Rec = recall, and FM=F-measure.

RETRACTED

## Data Availability

The authors have employed the dataset collected by the University of Queensland [12].
